# Associations Between Personality Functioning, Childhood Trauma and Non-adherence in Cardiovascular Disease: A Psychodynamically-Informed Cross-Sectional Study

**DOI:** 10.3389/fpsyg.2022.913081

**Published:** 2022-06-23

**Authors:** Karl Haller, Stefan Fritzsche, Irina Kruse, Grace O’Malley, Johannes C. Ehrenthal, Thomas Stamm

**Affiliations:** ^1^Department of Psychology, Brandenburg Medical School Theodor Fontane, Neuruppin, Germany; ^2^Department of Hematology, Oncology, and Tumor Immunology, Charité – University Medicine Berlin, Berlin, Germany; ^3^Agaplesion Bethanien Diakonie, Berlin, Germany; ^4^Cardiology Department, Schlosspark-Klinik, Berlin, Germany; ^5^Department of Pediatrics, Division of Oncology and Hematology, Charité – University Medicine Berlin, Berlin, Germany; ^6^Department of Psychology, University of Cologne, Cologne, Germany; ^7^Schloss Luetgenhof Hospital, Centre for Personal Medicine, Psychosomatics and Psychotherapy, Dassow, Germany

**Keywords:** adherence, cardiology, childhood trauma, personality functioning, psychodynamic, secondary prevention

## Abstract

**Objective:**

Although treatment adherence and lifestyle changes significantly improve the prognosis of cardiovascular disease, many patients do not comply with clinician recommendations. Personality functioning appears to be of importance and is hypothesized to be superior to symptom-based measures in explaining individual differences in non-adherence.

**Methods:**

194 cardiology inpatients (mean age = 70.6 years, 60% male) were assessed using self-report measures in a cross-sectional design. Patients were assessed using the short version of the Operationalized Psychodynamic Diagnosis Structure Questionnaire (OPD-SQS) to measure personality functioning, as well as the Childhood Trauma Screener (CTS), the Patient Health Questionnaire (PHQ-9) for symptoms of depression, and the Generalized Anxiety Disorder Scale-7 (GAD-7). To assess non-adherence we introduced a brief, novel scale.

**Results:**

Non-adherence correlated significant with personality functioning (*r* = 0.325), childhood trauma (*r* = 0.204) and depressiveness (*r* = 0.225). In a stepwise multiple regression analysis with socio-demographic variables inputted into the model, higher deficits in personality functioning, higher levels of childhood trauma, and male gender were associated with non-adherence (adjusted *R^2^* = 0.149, *F*_(3,190)_ = 12.225, *p* < 0.01). Level of depressive symptoms, anxiety, age, education, and income showed no significant additional predictive value and were excluded from the model.

**Conclusion:**

In cardiovascular disease, personality functioning, childhood trauma and male gender are associated with non-adherence and appear to be more important than symptom reports of depression and anxiety. This highlights the relevance of basic impairments in intra- and interpersonal functioning in chronic disease, where the patient’s adherence is central.

## Introduction

Cardiovascular disease (CVD) is a major cause of premature death and disability throughout the world (Smith et al., 2012). Although the medical understanding of CVD and its treatment options have improved significantly in recent decades, secondary prevention has shown to be an indispensable factor in reducing the risk of CVD and its negative consequences (Bansilal et al., 2015). Secondary prevention involves consistently taking one’s medication on a daily basis, and substantial changes in lifestyle. The World Health Organization (WHO) recommends smoking cessation and dietary changes such as the following: Salt reduction, eating at least 400 g of fruits and vegetables and a range of whole grains and pulses daily, at least 30 min of moderate physical activity a day, loss of weight or obesity, and considerably reducing one’s alcohol intake. Recommendations also include medical treatment of hypertension, high levels of cholesterol, fasting blood glucose and risks of thrombosis (World Health Organization, 2007). A large meta-analysis revealed that only about 50% of cardiovascular patients adhered to the medication prescribed to prevent myocardial infarction (Naderi et al., 2012). Another study which examined lifestyle factors such as regular physical activity, healthy diet, non-smoking, and moderate alcohol consumption meanwhile found that only approximately one third of the patients were adherent to all their advised restrictions and lifestyle changes (Huy et al., 2010).

Such strikingly poor rates of adherence are concerning given the strong evidence that lifestyle and medication adherence is closely linked to the occurrence of cardiological diseases and their course. In a systematic review and meta-analysis of prospective epidemiological studies, poor adherence to vascular medication was found to be responsible for roughly 9% of all CVD events in Europe (Chowdhury et al., 2013). According to this meta-analysis, good adherence could lead to a 20% lower risk of CVD and a 35% reduction of all-cause mortality. Further, a healthy lifestyle seems to be associated with a 66% reduced risk for cardiovascular disease (Barbaresko et al., 2018). Although there is clear proof of the importance of adherence to lifestyle recommendations for patients with CVD, changing patients’ behavior seems to be very challenging (McAlister et al., 2001).

The reasons for poor adherence are complex and diverse (Bosworth et al., 2011). Many studies emphasized the role of mental health in adherence, mainly focusing on patients with depression and anxiety (Bane et al., 2006; Gentil et al., 2012; Dempe et al., 2013; Kretchy et al., 2014; Gathright et al., 2017; Penninx, 2017). However, the role of psychiatric disorders in cardiology patients’ adherence seems to be intricate. Several studies indicate the negative influence of depression on adherence in CVD patients (Carney et al., 1995; Rieckmann et al., 2006; Casey et al., 2008; Berntson et al., 2015; Goldstein et al., 2017; Okunrinboye et al., 2019), although one study has highlighted that milder forms of depression may not necessarily be related to decreased levels of medication adherence (Okunrinboye et al., 2019). A range of mediators of this process have been proposed (Gellad et al., 2009; Manning and Bettencourt, 2011; Osborn and Egede, 2012; Hilliard et al., 2015) [e.g., social support (Osborn and Egede, 2012)]. The relationship between anxiousness and the likelihood of adhering to treatment recommendations seems even more ambiguous (DiMatteo et al., 2000). While some studies highlighted a link between anxiety and non-adherence (Bautista et al., 2012), others only found minimal associations (Schweitzer et al., 2007). The regular occurrence of severe panic attacks might lower the ability to follow prescriptions, but there is good reason to assume that moderate levels of anxiety might also increase the likelihood of following medical recommendations. This might especially be the case if anxious beliefs involve health-related issues (Bellg, 2004). These inconsistencies may not just be explained by severity of anxiety or depression, but also by other factors that define heterogeneity within a given psychiatric diagnosis, such as personality functioning or personality disorders (e.g., Köhling et al., 2015). Specific personality disorders as well as dimensional measures of levels of personality are related to health-related outcomes (Dokucu and Cloninger, 2019; Sinnaeve et al., 2021). Deficits in personality functioning appear to have a negative impact on disease progression and adherence (Collier et al., 1999) in mental illness (bipolar disorder (Wagner-Skacel et al., 2020; Ortelbach et al., 2022); eating disorders (Rohde et al., 2019); personality disorders (Zimmermann et al., 2014); major depressive disorder (Zeeck et al., 2020) as well as cancer (Wynn, 2010; Di Mattei et al., 2018) and chronic physical illness (Leichter and Dreelin, 2005; Pollock-BarZiv and Davis, 2005; Moran et al., 2007; Lee et al., 2010). Only two studies have examined the influence of personality disorders on non-adherence in cardiovascular health to date (Suárez-Bagnasco et al., 2015; Hall et al., 2019), indeed despite knowledge that personality disorders are an important risk factor for health-related matters such as physical functioning, role limitations, fatigue, and pain (Powers and Oltmanns, 2012). Furthermore, personality disorders are linked to several variables concerning general health status (Soeteman et al., 2008; El-Gabalawy et al., 2010).

The paucity of research on personality disorders on CVD patients’ treatment adherence may be explained by the low occurrence rates of severe personality disorders in this population (Pérez-Piñar et al., 2016). However, there is good reason to assume that milder impairments of basic personality functions, such as difficulties with emotion regulation, impaired social functioning and interpersonal problems, are more prominent in this cohort and also lead to serious problems of physical well-being and health-related behaviors (Bach and Hutsebaut, 2018; Nelson et al., 2018). As suggested by the Alternative Model for the Assessment of Personality Disorders (AMPD) of the DSM-5 (Bender et al., 2011) or the upcoming model for ICD-11 (Tyrer et al., 2019), general personality functioning in terms of basic self- and other-related emotion processing and regulation allow for the inclusion of subclinical impairments.

In addition to the more recent developments from formal psychiatric diagnosis, the concept of personality functioning has a long tradition in for example psychodynamic or interpersonal theory (Hopwood, 2018; Ehrenthal and Benecke, 2019), and describes biographically evolved and persistent patterns of emotion, cognition, regulation, and behavior. These patterns are shaped by early relational experiences (Zimmermann et al., 2012). Conveniently, the psychodynamic concept of ego integration offers scope for examining even milder forms of impairment in basic personality functioning, which, as discussed, may serve to clarify fundamental and important mechanisms underpinning problems in patient adherence (e.g., medication refusal and refusal to adopt lifestyle recommendations). Its role in predicting the course and symptom severity of physical illness, as well as its processing, also seems significant (Ehrenthal et al., 2019) and may be especially important in chronic diseases that demand a particularly high level of compliance and lifestyle changes.

In a similar vein, childhood trauma – which, theoretically, is closely linked to personality functioning (de Carvalho et al., 2015) – has been proposed as an important risk factor in CVD (Rozanski et al., 2005). While there is some evidence that childhood trauma has an impact on medication adherence in HIV (Mugavero et al., 2006; Whetten et al., 2013; Willie et al., 2016), to our knowledge, no research is available to date for CVD. However, it seems likely that exposure to adverse experiences such as sexual, physical, or emotional abuse in childhood could lead to difficulties in self-care such as implementing complex behavioral changes (Prather and Golden, 2009), and perhaps also to negative interactions with healthcare providers (Green et al., 2012).

The current study aims to address the research question as to whether deficits in basic intrapersonal and social functioning, defined as personality functioning, and a history of childhood trauma are associated with a higher self-reported tendency of non-adherence to secondary prevention guideline recommendations in cardiology inpatients. Furthermore, we aim to investigate whether personality functioning and a history of childhood trauma are better at predicting non-adherence than (a) more symptom-based variables such as depression and anxiety, as well as (b) basic socio-economic characteristics.

## Materials and Methods

### Study Design and Recruitment

Between May 2019 and March 2020, we recruited participants on two wards in the cardiological inpatient unit of the Ruppiner Kliniken, a general hospital in northeast Germany. Due to the focus on secondary prevention, only patients with a history of cardiological disease were included in the study. These patients were informed about the study and after providing informed consent, they were asked to complete a self-report assessment. Demographic information was also collected (namely age, gender, education, relationship status, income). Medical parameters such as medical diagnoses, including coronary heart disease, arterial hypertension, hyperlipoproteinemia and diabetes, were extracted based on file review. Inclusion criteria were a history of cardiological disease, at least 18 years of age, and completion of the questionnaire battery.

### Procedures

The local ethics committee of the Medical School Brandenburg – Theodor Fontane approved the study protocol.

### Measurements

#### Patient Health Questionnaire

The Patient Health Questionnaire (PHQ-9) is a 9-question, self-report depression subscale of the PHQ (Kroenke et al., 2001). Each item is based on the DSM-IV criteria for depression and the questionnaire can be used to predict the severity of depression. Patients are required to assess depressive symptoms (e.g., “feeling down, depressed or hopeless”) over the last 2 weeks on a 4-point Likert scale (where 0 = not at all and 3 = nearly every day). A total score ranging between 0 and 27 is achieved by adding all item scores. Values from 0 to 4 indicate none/minimal symptoms, 5 to 9 is considered mild, 10 to 14 is moderate, 15 to 19 is moderately severe, and 20 to 27 represents severe symptoms. In general, a cutoff score of 11 is considered indicative of severe depressive symptoms. A recent study by Kroenke, Spitzer and Williams showed good internal consistency (Cronbach’s α = 0.89/0.86) and construct validity compared with the 20-Item Short Form Health Survey (SF-20) questionnaire as well as good criterion validity (Kroenke et al., 2010).

#### Generalized Anxiety Disorder Scale-7

In order to assess anxiety we used the Generalized Anxiety Disorder Scale-7 (GAD-7), a self-report questionnaire for screening and measurement of the severity of generalized anxiety disorder (Spitzer et al., 2006). It forms part of the PHQ-D and is reported to also measure other anxiety disorders including social phobia, post-traumatic stress disorder and panic disorder (Kroenke et al., 2007). The GAD-7 consists of seven items reflecting states over the past 2 weeks (e.g., “feeling afraid as if something awful might happen”). The instrument contains a 4-point Likert scale (where 0 = not at all and 3 = nearly every day). Total anxiety scores range from 0 to 21 (0–4 = minimal, 5–9 = mild, 10–14 = moderate, 15–21 = severe). The internal consistency is reported to be good (Cronbach’s α = 0.92) and validity has been proven (Löwe et al., 2008).

#### The Operationalized Psychodynamic Diagnosis Structure Questionnaire

Personality functioning was measured according to the Levels of Structural Integration Axis (LSIA) of the Operationalized Psychodynamic Diagnosis (OPD-2) (OPD Task Force, 2008), a multiaxial psychodynamic diagnosis system which has attained wide usage in Germany in the last 20 years for both diagnostic and treatment planning purposes (Cierpka et al., 2007). The OPD covers five axes: Illness experience and treatment assumptions, relationships, mental conflicts, and personality structure, i.e., levels of personality functioning. We used the short form of the OPD Structure Questionnaire (OPD-SQS) (Ehrenthal et al., 2012; Ehrenthal et al., 2015), a 12-item screening instrument where item scores range between 0 and 4, for example: “Sometimes my feelings are so intense that I get scared,” “I sometimes feel like a stranger to myself,” or “I sometimes misjudge how my behavior affects others.” A total score is computed and ranges from 0 (“indicating high levels of personality functioning”) to 48 (“indicating notable impairment of personality functioning”), whereby lower scores represent lower personality functioning. The internal consistency (α = 0.89) and validity have been confirmed (Ehrenthal et al., 2012; Obbarius et al., 2019), and the long version also correlated with the expert ratings of the personality functioning to *r* = 0.62 (Dinger et al., 2014).

Beyond the use of the overall scale, the developers propose three subscales for research questions that are highly correlated with one other: self-perception, contact formation and relationship model (Ehrenthal et al., 2012). While the *self-perception* subscale links structural aspects of the self with emotion regulation skills, the *contact formation* subscale links interactional skills with aspects of self-uncertainty. Thirdly, the *relationship model* subscale maps the representation of relationship experiences which, accordingly, are associated with expectations for new relationships (Obbarius et al., 2019).

#### Childhood Trauma Screener

The Childhood Trauma Screener (CTS, Grabe et al., 2012) is a brief version of the Childhood Trauma Questionnaire (CTQ) (Bernstein et al., 1997; Bernstein et al., 2003; Wingenfeld et al., 2010), an internationally used, short self-assessment procedure for the retrospective recording of various traumas in childhood, including emotional, physical and sexual abuse as well as emotional and physical neglect. The CTS consists of 5 items scaled from 1 (not at all) to 5 (very often), whereby every item corresponds to one scale of the larger CTQ. The total score is built by adding the values of all items leading to a score ranging from 5 to 25. Studies have found good psychometric properties of the instrument with an internal consistency of α = 0.76 and correlation of *r* = 0.88 between the total sum score of the CTS and the CTQ (Grabe et al., 2012).

#### Measuring Non-adherence

Due to the lack of existing questionnaires that cover the desired range of non-adherence, we created a three-item scale. It was operationalized as a self-assessed overall tendency not to start recommended treatments, to not implement recommended lifestyle changes, and to discontinue recommended treatment, using a single item for each, respectively. The participants could rate their tendency on a 4-point Likert scale ranging from 1 (not at all) to 4 (very much). We calculated the total score and found a rather low internal consistency of Cronbach’s α = 0.55.

### Data Analysis

Statistical analysis and data preparation were carried out using IBM SPSS Statistics 27.

## Results

### Participants

While data was collected for 218 patients, due to missing data the final analyses was based on 194 participants. Table 1 reports the sociodemographic variables.

**TABLE 1:** Characteristics of the participants in the study.

	*n*	(%)	*M*	(SD)
Gender – male – female	115 79	59.3 40.7		
Age (years)			70.64	(11.77)
Family status – single – partnership	65 129	33.5 66.5		
Number of children			1.93	(0.97)
Years of education			14.28	(2.82)
Profession status – working – retired – other	33 151 10	17.0 77.8 5.2		
Net income (in euros per month) – less than 500 – 500–1000 – 1000–2000 – 2000–3000 – 3000–5000 – more than 5000	4 53 101 22 9 5	2.1 27.3 52.1 11.3 4.6 2.6		

*N = 194.*

Table 2 presents the information regarding the participants’ somatic functioning and medical diagnoses. Limited information regarding mental illness was obtained from the file review. For this reason, we report the number of participants which had severe depressive symptoms based on the PHQ-9 [cut-off score of ≥11 as recommended by Gräfe et al. (2004)].

**TABLE 2:** Diagnosed illnesses and psychometrics properties of the participants in this study.

	*n*	(%)	*M*	(SD)
**Illness**				
Coronary heart disease (CHD)	138	71.1		
CHD mainstem stenosis	16	8.2		
Myocardial infarction	44	22.7		
Heart failure	66	34.0		
Cardiac decompensation	15	7.7		
Cardiac arrhythmia	57	29.4		
Arterial hypertension	168	86.6		
Severe depressive Symptoms (PHQ-9 ≥ 11)	53	27.3		
**Psychometric total score (range)**				
Non-adherence (0–4)			1.56	(0.55)
PHQ-9 (0–27)			7.54	(5.08)
GAD-7 (0–21)			4.86	(3.97)
OPD-SQS (0–36)			10.76	(7.48)
CTS (5–25)			8.00	(3.24)

*PHQ-9, Patient Health Questionnaire; GAD-7, Generalized Anxiety Disorder Scale-7; OPD-SQS, OPD Structure Questionnaire, CTS, Childhood Trauma Screener.*

*N = 194.*

As summarized in Table 2, overall participants endorsed agreeing to implement recommendations. Overall, levels of depression and anxiety were mild in our participant group. Indeed, personality functioning as indicated by the OPD-SQS was generally in the low range indicating relatively high levels of personality functioning.

To examine whether the group of the 24 excluded participants differed significantly from the 194 included patients in the reported variables, *t*-tests and chi-square tests were conducted. Participants that were excluded due to missing data differed significantly in the frequency of CHD (94% in the excluded group vs 71% in the included group; *p* = 0.027). All other variables showed no significant differences.

### Statistical Analysis

We hypothesized, and found evidence of, a statistically significant, positive relation between personality functioning (OPD-SQS) and non-adherence (*r* = 0.325, *p* < 0.001). Also, depressiveness and childhood trauma, respectively showed small but significant correlations with non-adherence (*r* = 0.225, *p* < 0.001); (*r* = 0.204, *p* < 0.001). According to conventional models of *p*-values, generalized anxiety was not significantly associated with self-reported non-adherence (*r* = 0.140, *p* < 0.051). To test for the influence of socio-demographic variables, we also included age, years of education and net monthly income, and found no connection to non-adherence. In addition, to control for possible gender differences, we conducted a *t*-test. The level of non-adherence differed statistically significant for men and women, *t*_(192)_ = 2.095, *p* < 0.05.

Stepwise multiple regression analysis was used to test if the reported variables significantly predict participants’ self-reported non-adherence. Table 3 shows the regression models with the three steps of variable inclusion. Model 3 indicates that the three predictors explained 14.9% of the variance (Adjusted *R*^2^ = 0.149, *F*_(3,190)_ = 12.225, *p* < 0.01). It was found that levels of personality functioning (OPD-SQS) significantly predicted non-adherence (β = 0.33, *p* < 0.001), as did extent of childhood trauma (CTS) (β = 0.17, *p* < 0.05) and gender (β = −0.19, *p* < 0.05). Depressiveness (PHQ-9), generalized anxiety (GAD-7), age, years of education and net income showed no significant additional predictive value and were thus not considered any further for the model.

**TABLE 3:** Summary: predicting non-adherence in linear stepwise regression analysis.

	β	*p*	*F*	*R* ^2^_*adj*_	Δ*R*^2^
**Model 1**		0.000**	***F*_(1,192)_ = 22.609**	**10.1**	**0.105**
**OPD-SQS**	**0.325**	0.000**			
GAD-7	−0.63	0.449			
PHQ-9	0.095	0.218			
CTS	0.145	0.036*			
Gender	−0.17	0.013*			
Age	0.038	0.548			
Net income	−0.25	0.712			
Years of education	−0.013	0.849			
**Model 2**		0.000**	***F*_(2,191)_ = 14,778**	**12.5**	**0.029**
**OPD-SQS**	**0.335**	0.000**			
**Gender**	−**0.17**	**0.076**			
GAD-7	−0.048	0.560			
PHQ-9	0.105	0.167			
CTS	0.172	0.013*			
Age	0.063	0.360			
Net income	−0.065	0.346			
Years of education	−0.60	0.394			
**Model 3**		0.000**	***F*_(3,190)_ = 12,225**	**14.9**	**0.28**
**OPD-SQS**	**0.302**	0.000**			
**Gender**	−**0.192**	0.005**			
**CTS**	**0.172**	0.013*			
GAD-7	−0.044	0.584			
PHQ-9	0.110	0.142			
Age	0.077	0.257			
Net income	−0.065	0.341			
Years of education	−0.071	0.305			

PHQ-9, Patient Health Questionnaire; GAD-7, Generalized Anxiety Disorder Scale-7; OPD-SQS, OPD Structure Questionnaire; CTS, Childhood Trauma Screener. b = Standardized regression coefficient; R^2^_adj_ = adjusted R-squared; ΔR^2^ = difference in the proportion of variance explained. Bold variables indicate inclusion in the model. N = 194, *p < 0.01, **p < 0.001.

To investigate the relationship between personality functioning and self-reported non-adherence in more detail, we also calculated the subscales of the OPD-SQS. Internal consistency of all three subscales was acceptable with Cronbach’s α ranging from.685 to.699. Correlational analysis revealed small to moderate associations with non-adherence for all three subscales (self-perception, *r* = 0.213, *p* < 0.01); (contact formation, *r* = 0.267, *p* < 0.001); (relationship model, *r* = 0.305, *p* < 0.001).

## Discussion

In our sample of 194 cardiology inpatients, stepwise multiple regression revealed personality functioning and childhood trauma as significant predictors of non-adherence. In contrast, levels of depression and anxiety were not predictive of non-adherence. 10% of the variance could be explained by levels of personality functioning alone (Adjusted *R*^2^ = 0.101, *F*_(1,192)_ = 22.609, *p* < 0.001). When controlling for sociodemographic variables such as age, gender, net income, and years of education, only gender had a significant association with non-adherence with males identified as more likely not to comply with treatment recommendations. A lower level of personality functioning on the OPD-SQS, higher levels of childhood trauma, and male gender, were predictive of higher levels of non-adherence, explaining 15% of the variance in scores.

In addition, symptoms of depression and to a certain degree anxiety were observed to correlate with non-adherence, which is in line with previous studies (Ziegelstein et al., 2000; Kuhl et al., 2009). In our sample, anxiety showed a weaker, non-significant association with non-adherence compared with the results for depression. This could be explained by differences in prototypical psychopathology (World Health Organization, 2004). While anxiety is characterized by symptoms such as increased activation and agitation, depressive symptomatology is usually characterized by symptoms such as lack of motivation, low energy, limited ability to concentrate, and pessimistic beliefs about the future. As such, typical depressive symptoms are likely to be more related in content to non-adherence than those of anxiety. All the same, the clearest association occurred with personality functioning predicting non-adherence in the regression model. This finding is in support of our proposal that fundamental psychological features and abilities, as conceptualized in the framework of personality functioning (Ehrenthal et al., 2015), may play an essential role in adhering to lifestyle-related medical recommendations.

Which particular aspects of personality functioning are relevant in the context of non-adherence to chronic cardiac disease may be an important focus for future research. In our study, aspects of self-perception, contact formation, and relationship model had a significant positive correlation with non-adherence. The strongest correlation was shown with the relationship model subscale (*r* = 0.305), which points to the centrality of early shaped relational patterns in informing non-adherence; most likely played out in the clinician-patient relationship. Non-adherence most likely occurs against the backdrop of an interactional, relational event. On the OPD-SQS, the relationship dimension of personality functioning primarily maps the tendency of people to experience contact with others as threatening and uncontrollable (Ehrenthal et al., 2012). It is plausible therefore that such a personality effect could influence willingness or ability to make and uphold behavioral adaptations, whereby subclinical difficulties in experiencing the other person as trusting and helpful may lead to an increased tendency not to implement or to discontinue treatment recommendations. Accordingly, clinical implications of this may include scope for cardiologists to assess patient personality functioning earlier in treatment planning. This may enable clinicians to identify negative personality effects on adherence early and intervene appropriately, e.g., by lining up further multidisciplinary supports and liaising with psychology, psychosomatic medicine and psychiatry (Sudhir, 2017). In this vein, some possibilities may include providing training to clinicians on how to interact with such patients fruitfully, such as how to focus on problem behaviors without punishing; to involve mental health professionals at an early stage of treatment; to adopt regular staff meetings to liaise regarding patients; and to establish realistic expectations regarding patients’ capacity to implement their healthcare recommendations and indeed support them in achieving them (Peteet et al., 2011). In addition, several psychodynamic treatment approaches to enhance personality functioning have been developed (Kernberg et al., 2008; Bateman and Fonagy, 2013; Rudolf, 2020). Initial attempts have been made to implement such psychotherapy techniques to support adherence in the context of medical recommendations for chronic conditions by promoting a more accurate understanding of their mental state (Malberg, 2019). Further research is needed to derive more specific treatment recommendations from this.”

Our findings suggest that people who suffered trauma in childhood also have more difficulty adhering to medical recommendations. Several studies have shown that people with childhood trauma are more likely to develop insecure attachment styles, which are associated with difficulties in seeking help and maintaining stable relationships (Pearlman and Courtois, 2005; Clark et al., 2011; Millar et al., 2021) and other factors related to somatic medicine (Graetz et al., 2013; Graf et al., 2020; Graetz et al., 2021). Therapeutic alliance, a marker of a stable relationship, indeed appears to play an important role in adherence (Pringle and Fawcett, 2017). Individuals with a history of childhood trauma may be more likely to encounter challenges in trusting others, including their medical caregivers. Our findings point toward the value in identifying childhood trauma among CVD patients. In case of a trauma history, appropriate relational and rapport-based adjustments may be made to the clinical course, e.g., longer appointment durations during early treatment to facilitate trust, or the application of a greater focus on a person-centered approach.

Our results indicated that men tended to report higher levels of non-adherence than women. Interestingly, this contradicts other study findings on the role of gender in adherence (Vervloet et al., 2020), with several studies and reviews finding women to be more non-adherend to statins (Lewey et al., 2013; Ofori-Asenso et al., 2018; Ingersgaard et al., 2020), or indeed no such gender differences (Holmes et al., 2012; Holt et al., 2013). It seems likely that differences in medication adherence might be explained by variation in side effects, beliefs about drugs, and treatment recommendation by physicians (Vervloet et al., 2020). In contrast to medication adherence, women seem to be more willing to change their lifestyle (Jarbøl et al., 2017). This might explain why we found men to report higher levels of non-adherence, as we asked regarding the general tendency not to start recommended treatments, implement recommended lifestyle changes, and to discontinue recommended treatments. Our results highlight the general assumption in cardiology that gender differences in symptomatology, treatment options, adherence and perception by medical staff should be heeded and researched further (Möller-Leimkühler, 2007; Mosca et al., 2011; Goldstein et al., 2016).

In interpreting the findings of this study, we note several limitations. All variables were measured using self-report, and accordingly may be subject to recall bias or social desirability. All the same, in the case of non-adherence at least, the influence of social desirability on self-reported adherence has been proposed to be overestimated (Wagner and Miller, 2004). Several alternative approaches to measuring non-adherence have been developed (Vitolins et al., 2000), however, most are limited to assessing adherence to medication (e.g., electronic medication packaging (EMP) devices or medication counts) (Kronish et al., 2021). Other measurement methods directly capture clinical outcomes as an indicator of non-compliance, but are proposed to be confounded by various individual and disease-specific factors (Nguyen et al., 2014). As such, when it comes to identifying subjective burden of adhering to a large variety of different treatment recommendations, self-assessment appears to be a reliable and valid measurement approach, especially when it comes to identifying patient burden and their associated support needs. A reasonable approach for future research may therefore be to balance self-report scales with behavioral measures, such as nutrition or exercise diaries, that counteract possible recall biases (Nguyen et al., 2014; Anghel et al., 2019). The measurement of childhood trauma may also have been influenced by recall bias. Our sample is comparatively old (mean age = 70.6 years) and it is conceivable that memories of abusive experiences in childhood are biased due to cognitive impairment. We did not examine the patients for cognitive impairment ourselves but screened the patient files for clinical diagnosis and found no case of dementia or mild cognitive impairment in our sample. However, we acknowledge that it is possible that these diagnoses have been overlooked by cardiology colleagues. While we cannot completely rule out a possible recall bias, retrospective recording of ACEs seem comparatively reliable (Brewin et al., 1993; Hardt and Rutter, 2004) and has also been used in other studies with participants of advanced age (Felitti et al., 1998).

We note that our sample reported good overall personality functioning, with low personality functioning presenting rarely. However, this finding may be considered representative of the cardiology patient group as a whole. In comparison with other studies the picture that emerges is that the degree of mental illness seems to be related to the level of personality functioning. For example, diabetic patients show better scores in personality functioning (Ehrenthal et al., 2019) than patients who were in outpatient treatment for mental illness (Ehrenthal et al., 2012) and these in turn show better scores than patients who were in inpatient treatment for mental illness (Obbarius et al., 2019). We caution that a conclusive evaluation of personality functioning on the OPD-SQS is best achieved when conducted by a trained clinician as opposed to by self-report. This was beyond the scope of this study. However, on the basis that sufficient agreement between self-assessment and expert rating has been demonstrated (Dinger et al., 2014), we consider this self-report measure to have had good and sufficient reliability and validity overall.

Finally, although the psychodynamic concept of personality functioning makes theoretical assumptions about the early childhood development of these traits (Dagnino et al., 2020; Krakau et al., 2021), due to the cross-sectional design of the study we cannot make a clear statement about the causality of the associations between personality functioning and non-adherence. However, we collected data from a large and well-characterized clinical sample which serves as an important and appropriate first step in investigating associations between these variables. Future research should attempt to unpick a potential causal relationship and adopt a longitudinal design: For example, in investigating to what extent the level of personality functioning at initial diagnosis of a cardiological disease can predict the implementation of recommended medical measures across the treatment and clinical course. Another interesting question would be how stable personality functioning is over time. To examine these temporal relationships more closely would be an intriguing line of inquiry. Indeed, there are initial findings that show that the OPD-SQS is also suitable for measuring change in the context of psychotherapeutic treatment (Lübke et al., 2021).

## Conclusion

Our findings highlight the role of personality functioning and trauma as important predictors of treatment adherence in cardiovascular disease, indeed to a greater extent than psychopathology symptoms (depression, anxiety) and demographic factors. The relevance of discrete and fundamental personality features, and their role in intra- and interpersonal functioning as reflected in the patient and care provider relationship, may be important in informing cardiological care given the centrality of lifestyle changes in preventative medical care and management of cardiovascular disease.

## Data Availability Statement

The raw data supporting the conclusions of this article will be made available by the authors, without undue reservation.

## Ethics Statement

The studies involving human participants were reviewed and approved by the Ethics Committee of the Medical School Brandenburg Theodor Fontane. The patients/participants provided their written informed consent to participate in this study.

## Author Contributions

KH, SF, IK, and JE contributed to the conception or design of the work. KH, SF, IK, and TS contributed to the acquisition and analysis or interpretation of data for the work. KH and SF drafted the manuscript. GO’M, TS, and JE critically revised the manuscript. All authors contributed to the article and approved the submitted version.

## Conflict of Interest

SF was employed by the company Agaplesion Bethanien Diakonie. The remaining authors declare that the research was conducted in the absence of any commercial or financial relationships that could be construed as a potential conflict of interest.

## Publisher’s Note

All claims expressed in this article are solely those of the authors and do not necessarily represent those of their affiliated organizations, or those of the publisher, the editors and the reviewers. Any product that may be evaluated in this article, or claim that may be made by its manufacturer, is not guaranteed or endorsed by the publisher.
